This article has been retracted.

# Establishment, Analysis, and Application of the Information Transmission and Response Model for Students of Vocational Colleges under Public Health Emergencies

**DOI:** 10.1155/2022/6701364

**Published:** 2022-01-06

**Authors:** Hengliang Chen, Zilin Li, Fei Luo

**Affiliations:** ^1^Shenzhen Institute of Technology, Shenzhen 518116, China; ^2^Department of Mechanical Engineering, Tsinghua University, Beijing 100084, China; ^3^Faculty of Education, Mahasarakham University, Maha Sarakham 44000, Thailand

## Abstract

To provide a basic quantitative mathematical model for data analysis, decision-making support, and application of information systems oriented to emergency research, this paper established an information transmission response model for school students under such system mathematically based on actual school information transmission data during COVID-19 prevention. This paper proposes an emergency information management method—a two-step emergency information management method. It can be referenced for promotion of the development of IT-based school management, enhancement of IT application in school emergency information management, and improvement of the speed and accuracy of information transmission.

## 1. Introduction

Novel coronavirus disease (COVID-19) that broke out at the end of 2019 has the significant features of high abruptness, strong infectivity, and broad prevalence and is a sudden test for governments, enterprises, and schools. As social organizations with a high level of aggregation, schools need to acquire accurate information on all teachers and students quickly and accurately and make decisions at the right time, which is particularly important. Accordingly, it is of urgent realistic significance to conduct an information management study on public health emergencies and improve the timeliness of information acquisition and decision making.

Emergencies usually refer to sudden events which are difficult to be predicted and prevented [1], such as a public health emergency that occurs suddenly and may cause a massive health damage. COVID-19 is a typical public health emergency. In information management of emergency response, the key to emergency response capacity is ensuring information accuracy and improving information response speed. Only if an efficient public health emergency response information system is established can quick, accurate, and comprehensive information be provided to decision makers, thus ensuring that crisis response decisions are accurate and effective [2]. During the management of vocational college students, it is necessary to master students' trips and health status timely, accurately, and completely [3, 4]. This paper establishes a school information transmission response model for emergency information management and discusses the characteristics and response pattern of information transmission by collecting and analyzing epidemic data of vocational college students [5–7].

## 2. Information Transmission System Architecture under COVID-19 Outbreak

### 2.1. Organizational Structure of Information Transmission

As shown in Figure 1, the organizational structure of information transmission under public health emergencies during information management of vocational college students is divided into three parts, which are the data acquisition system, data storage and analysis system, and application and output system, as detailed in the following:

1. The data acquisition system acquires basic data, such as basic information, health status, and trip information of students in this event, usually reported by students.
2. The data storage and analysis system stores and encodes basic data. For example, class advisors, counselors, and supervisors compile and store basic data and transfer it to the system of the next level. Normally, it includes three levels of responsibility of level of class advisors, counselors (or information administrators), and supervisors. In the student management system of Chinese vocational colleges, the head teacher is mainly the grass-roots manager, mainly responsible for the daily management of the class, generally managing 30–50 students. Counselors are mainly responsible for the student management of a department, who work for head teachers, students, and managers. Generally, there are 300–500 students with 2–3 counselors. The supervisor is generally the deputy director of a department, responsible for the daily work of students in a department, mainly for class advisors and counselors. Generally, there is one supervisor in a department.
3. The application and output system makes decisions on encoded information, feeding it back to management work and generating an output for transmission to management at the next level. This is usually the responsibility of decision makers.

### 2.2. Contents and Characteristics of Information Transmission

Contents acquired for information transmission (sampling) are namely transmitted data. In this paper, transmitted contents under COVID-19 mainly include basic information, trip information, and health status information of students, as shown in Table 1.

When COVID-19 is a public health emergency and schools are important public places, the information transmission characteristics are as follows:

1. Students are aged 15–22 years, three-/four-year students from senior high schools are aged 17–22 years, and five-/six-year students from junior high schools are aged 15–21 years
2. Students are mentally immature, have highly flexible personalities and a strong curiosity for new things, and like new communication modes (e.g., WeChat, microblog, and short video)
3. Information transmission is highly time bound, and such information should usually be submitted and closed daily to master student information in real time
4. Information contents are highly accurate, where information for public emergencies should be 100% accurate, and any error may result in major damages and losses
5. Information contents are discrete

### 2.3. Network Architecture of Information Transmission

In the 1940s, Shannon proposed a communication system model and defined information source, channel, and destination. It can be seen from the characteristics of information transmission of vocational college students under COVID-19 outbreak that the network architecture for information transmission is as shown in Figure 2.

1. The network nodes are A, B, and C, which correspond to the data acquisition system, data storage and analysis system, and application and output system shown in Figure 2, respectively.
2. Information channels are divided into permanent and temporary information channels. Permanent information channels are denoted by the solid lines in Figure 2 and represent paths that must be gone through by information transmission, such as information transmission from A to B and from B to C in a class group in the form of broadcast by means of WeChat or a QQ group; temporary information channels are denoted by the dotted lines in Figure 2 and represent information channels built temporarily once it is found that information has to be further confirmed during transmission to collect temporary information. In this model, node A and B are responsible for the collection, analysis, and transmission of basic data, and node C is responsible for the external output of information. The information transmission between node A and B are bidirectional. Node C is a unidirectional external output from the node B, and there is no direct connection between A and C. For example, some special data in this pandemic need to be collected through temporary communication with students by counselors and supervisors, such as “one-to-one” telephone communication.

## 3. Information Transmission Response under COVID-19 Outbreak

### 3.1. Information Sampling Results

To ensure the timeliness and accuracy of information transmission in school emergency information management under COVID-19, the information sampling results are as follows [8–11]:

1. Time: from February 5 to April 3, 2020, daily reporting.
2. Sample: electromechanical discipline, aged 16–22 years, 1,531 persons.
3. Class response statistics: such statistics include each student's admission year, discipline information, class information, academic system, and daily information response data, as shown in Table 2. The overall response is shown in Figure 3.

### 3.2. Establishment of an Information Transmission Response Model

#### 3.2.1. Deweighting of Information Transmission Response

As shown in Figure 4, there are two peaks in overall response including 0:00 and 10:00. It can be seen that the surveyed response data have been superimposed by the weighted activity data arising from the student daily routine, and it should be deweighted when the response model is established [12].

The deweighting of the overall response is shown in Figure 5.

- There are still two peaks after deweighting, where response peak 3 at 0:00 is elevated relative to the predeweighting level, and response peak 4 at 10:00 is much reduced, eliminating the impact of most of the online activity significantly.
- However, the response peak at 10:00 remains. The response peak at 10:00 remains because the WeChat activity curve is not accurate enough, e.g., including night activity data of overseas users; second, students would replenish information that should have been confirmed earlier when they wake up in the morning, resulting in a subjective small peak; third, except the small peak around 10:00, the whole response process drops monotonically, and the longer the time is, the closer the response proportion is to 0%.

#### 3.2.2. Establishment of an Information Transmission Response Model

It can be seen from the deweighted information transmission response that the information transmission response model can be data fitted with an exponential function, namely, *y*=*a* · *e*^−*bx*^. The built-in curve fitting tool of MATLAB is used for curve fitting, and an enhanced algorithm based on the nonlinear least square method plus least absolute residual (LAR) is used. The fitting model is *y*=0.4103 · *e*^−0.7066*x*^.

It can be seen from the model calculation results in Figure 6 and the overall data fitting chart in Figure 7 that

1. The standard deviation (RMSE) is 0.00823
2. The determination coefficient *R*-square is 0.992; i.e., this model highly coincides with the actual survey results
3. It is verified that the model can fit the response distribution very well by comparing the fitting curve with the actual response distribution curve

### 3.3. Verification of the Information Transmission Response Model

#### 3.3.1. Verification of Effectiveness

It can be seen from Figures 8 and 9 that when the student response curves in the two dimensions of student age structure and discipline structure are compared with the fitting model, all students of different admission years and disciplines coincide well with the fitting model, proving that the fitting model is effective.

#### 3.3.2. Repeatability Verification

To verify the repeatability of the model, the same information transmission structure and mode and sampling contents are used, and the sampling time is adjusted, namely, changing the information release time to after 9:00 a.m., for a seven-day experiment. The results are as shown in Figures 10–13.

It can be seen from Figures 10–13 that the response chart after time adjustment still fits the calculation model very well, the transmission response coefficient remains unchanged at 0.7066, and the overall information response will not change significantly, proving the repetition of the fitting model. On the other hand, a significant deviation occurs on the response curve between 9:00 and 11:00 and coincides with the small peak during the same time period before the sampling time adjustment, indicating that the actual user activity leads to the result difference, and the WeChat user activity data in the literature will create a certain deviation as the reference.

### 3.4. Methodology for Characteristic Values of the Information Transmission Response Model

It can be seen from Section 3.3 that the depiction of such information from transmission to confirmation by the exponential function has a high fit, and *a* · *e*^−*bt*^ may be used to denote the number of persons responding within hour *t* after information release.

It is integrated to obtain the total number of persons responding after *t* hours of information release. If it is assumed that *g*(*t*) is the proportion to the total number of persons and *g*(*t*)=1 when *t*⟶*∞*, it can be seen that *g*(*t*) is

(1) $$\begin{array}{c} g\left(t\right)=1-e^{-ct}, \end{array}$$

where *g*(*t*) is the overall response proportion after information release; *c* is the transmission response coefficient and denotes the rate of information transmission. For *c*=0.7066 in the model as mentioned in this paper, the proportion to the total number of persons of this model is *g*(*t*)=1 − *e*^−0.7066*t*^. The curve and the variation pattern are shown in Figure 14 and Table 3.

*f*(*t*) is used to denote the response proportion within hour *t* ~ *t*+1 after information release, and the following is obtained:

(2) $$\begin{array}{c} f\left(t\right)=\left(1-e^{-c}\right)\cdot e^{-ct}. \end{array}$$

The response proportion within the first hour after information release is obtained from the function *f*(*t*); i.e.,

(3) $$\begin{array}{c} c=-\ln\left[1-f\left(0\right)\right]. \end{array}$$

If *g*(*t*)=1 − *e*^−*ct*^ denotes the total amount of response, *h*(*t*)=*e*^−*ct*^ denotes the total amount of nonresponse. However, the prerequisite to this model is that the activity of all people in each hour is the same, while data will change under the actual activity curve. It is inadvisable to calculate a new *f*′(*t*) as the actual response proportion by multiplying the activity index by *f*(*t*) because the overall response (proportion) *g*(*t*) is then not equal to 100% under such condition.

To solve this problem, *V*(*T*) is used to denote the user activity under each moment, and then, the actual response proportion *f*′(*t*) is

(4) $$\begin{array}{c} f{}^{\prime }\left(t\right)=m\cdot V\left(T+t\right)\cdot \left(1-e^{-c}\right)\cdot e^{-ct}, \end{array}$$

where *T* denotes the actual time, namely, hour of day; *t* denotes the duration of information release; *V*(*T*) denotes the user activity at the current moment; and *m* is the ratio correction factor. The overall response *g*′(*t*) is

(5) $$\begin{array}{c} g{}^{\prime }\left(t\right)=m\cdot \sum_{i=0}^{t}\left[V\left(T+i\right)\cdot \left(1-e^{-c}\right)\cdot e^{-ci}\right]. \end{array}$$

In case of *g*′(*∞*)=1, it follows that *m*=1/∑_*i*=0_^*t*^[*V*(*T*+*i*) · (1 − *e*^−*c*^) · *e*^−*ci*^].

There is a simpler way here to determine the value of *m*. Without regard to activity, the response proportion data in the first hour alone can be used to calculate the transmission response coefficient; with regard to activity, the data of the first two hours *f*′(0) and *f*′(1) can be used to calculate the transmission response coefficient and the ratio correction factor comprehensively. *f*′(0) is divided by *f*′(1) to obtain the following value:

(6) $$\begin{array}{c} \frac{f{}^{\prime }\left(0\right)}{f{}^{\prime }\left(1\right)}=\frac{V\left(T\right)\cdot e^{c}}{V\left(T+1\right)}. \end{array}$$

The transmission response coefficient *c* can be calculated from the abovementioned formula and, therebym the ratio correction factor *m*.

In sum, this model can predict information transmission response curves under different activities quite completely.

## 4. Application of the School Information Transmission Response Model to the Emergency Information Management of Vocational Colleges

 *h*(*t*)=*e*^−*ct*^ denotes the total amount of nonresponse. There is a very interesting point here; i.e., if the information transmission mode (namely, the transmission response coefficient *c*) is not changed and information transmission is conducted again in the same way several hours after the first information transmission, the overall transmission curve will not be affected in any way. Therefore, repeated information release has little impact on the whole information transmission process; i.e., the rapidity of WeChat communication fails when it reaches a certain stage. To ensure that all people complete information receiving as soon as possible, we have to conduct customized information release for those not responding several hours after release, and the specific time point depends on the total number of people and the information transmission mode.

### 4.1. Application of the Emergency Information Management Workflow

It can be seen from the information transmission response model that emergency information management includes scheme establishment and arrangement, data acquisition and analysis, information transmission response model establishment, and emergency management decision making, as detailed in the following.

#### 4.1.1. Scheme Establishment and Arrangement

This includes establishing an emergency management working scheme and assigning tasks, in which the establishment of an emergency management working scheme includes the establishment of working requirements, scope of work, schedule, and staffing and supporting arrangements; assigning tasks including releasing the time, scope of information sampling, person responsible for information transmission, and total number of persons of information sampling; and setting the scheme completion time *t*_complete_.

#### 4.1.2. Data Acquisition and Analysis

To ensure quick and accurate data acquisition in emergency information management, the two-step acquisition method is used to acquire sampling information. In the first step, information is transmitted from A to B and from B to C in a class group in the form of broadcast by means of WeChat or a QQ group; in the second step, information is transmitted from A to B and from B to C by means of “one-to-one” mobile phone or telephone communication.

#### 4.1.3. Information Transmission Response Model Establishment

This is divided into two stages, namely, calculating the characteristic values of the information transmission response model and drawing a transmission model curve to predict information.

First, we calculate the characteristic values of the transmission response model. The proportion of persons completed is calculated one hour after information release to calculate the transmission response coefficient *c* and the correction factor *m*, such as  *c*=0.7066 and correction factor *m* obtained in the experiment in this paper. It can be seen that the overall information response curve without regard to the second stage is as in Figure 15.

Second, we draw a transmission model curve to predict information. The switching time of one-to-one telephone confirmation is calculated according to the completion time point of information sampling and the characteristic values of the transmission model. The *t* obtained by solving the equation 1 − *e*^−*ct*^=1+*k*(*t* − *t*_complete_) is namely the planned communication scheme switching time *t*_switching_.

#### 4.1.4. Emergency Management Decision Making

Emergency management decision making includes predictive decision making, completing the information transmission task, and conclusive decision making. Predictive decision making is making the earlier implementation of decision making possible in case of an emergency based on the response feedback of the prediction curve; the information transmission task will be completed at *t*_complete_ by conducting information transmission from A to B and from B to C for those not responding by means of “one-to-one” mobile phone or telephone communication at the preset switching time *t*_switching_; conclusive decision making is giving feedback on the finally acquired information and the predictive decision.

### 4.2. Analysis of the Emergency Information Management Method

To determine the accurate time of completion of the whole process, we performed a simulation test on this method. It is assumed that the volume of one-to-one telephone communication per unit time is constant, so it can be inferred that its response variation is linear [13]. The defined direct confirmation coefficient *k* denotes the proportion of people that can be confirmed for information directly by telephone per unit time and is expressed in percent per hour. The magnitude of the direct confirmation coefficient *k* depends on the human resource input and the total volume of confirmation.

To determine the starting time of one-to-one telephone communication, the proportion of completion of stage 1 needs to be set and can be calculated by *g*(*t*)=1 − *e*^−*ct*^. If telephone communication is set to begin at 90% of completion, the calculated starting time is 3 hours 15 minutes after information release; if the set proportion is 95%, the starting time is 4 hours 14 minutes; and if the set proportion is 98%, the starting time is 5 hours 32 minutes. The corresponding response curve is shown in Figure 16.

In this model, it is assumed that the direct confirmation coefficient *k*=15%/*h*. It can be seen from Table 4 that, for different proportions of completion in stage 1, the starting and ending times in stage 2 can be calculated. It can be seen that if the proportion is set lower, more time will be needed in stage 2, but the advantage is that the whole transmission process of information release can always be completed faster. When information transmission response is slow in the late stage, the double confirmation method can shorten the information transmission period effectively, which is a necessary measure in the whole information transmission process.

## 5. Conclusions

In conclusion, this paper studies the information transmission system and its response in public health emergencies (e.g., COVID-19), including the following:

1. It analyzes the organizational structure, network architecture, transmission process, and transmission mean of the information transmission system in school emergency information management under COVID-19 outbreak
2. It establishes the information transmission response model and discusses how to calculate its characteristic values
3. It tests the information transmission response model and proves that the curves in two dimensions well coincide with the fitting curve
4. It establishes the emergency information management workflow and analyzes the actually used key parameters, such as the completion time of information sampling, the resource input, and the relationship between the time points of switching between two information transmission modes
5. The information transmission response model can be applied to social organizations with similar information transmission structures and modes, such as schools, enterprises, and public institutions

In future research, we intend to study the information transmission and corresponding models under different group activity laws and different application scenarios, such as the impact of actual students' WeChat activity laws and course selection activities on the model. Then, we would study how to improve the corresponding efficiency and accuracy, such as the impact of the reward and punishment mechanism, time sharing, and batch intervention on the model.

## Figures and Tables

**Figure 1:** Organizational structure for information transmission.

**Figure 2:** Network architecture of information transmission.

**Figure 3:** Statistics of overall student information response.

**Figure 4:** WeChat-based time-shared activity chart.

**Figure 5:** Distribution of information response after deweighting.

**Figure 6:** Model calculation results.

**Figure 7:** Overall data fitting chart.

**Figure 8:** Comparison between response and fitting curves of students of different grades.

**Figure 9:** Comparison of response and fitting curves of different disciplines.

**Figure 10:** Comparison between the fitting chart and overall data deweighted response curve.

**Figure 11:** Comparison between response and fitting curves of students of different grades.

**Figure 12:** Comparison of response and fitting curves of different disciplines.

**Figure 13:** Comparison between overall response change (after deweighting) and fitting curve.

**Figure 14:** Variation of overall response to student information.

**Figure 15:** Overall information response curve (reference).

**Figure 16:** Response variation curve based on the two-step method.

**Table 1:** Contents transmitted.

Type	Content
Basic information	Name, gender, identity, phone number, class, class advisor
Trip information	Time of staying in or passing through Wuhan, time of staying in or passing through Hubei, current location, planned time of returning to Guangdong
Health status information	Date of abnormal clinical symptom, date of going to hospital, date of home observation, date of intensive observation, date of suspected case, date of release of medical observation, date of confirmed diagnosis, time and date of contact with a patient

**Table 2:** Response in statistical form of each class.

Date	Class	Proportion of system declaration (unit: minute)								
		60	120	180	240	300	360	420	480	—
										

**Table 3:** Time-shared table of overall response to student information.

Number of hours	Overall response (%)	Number of hours	Overall response (%)	Number of hours	Overall response (%)
1	50.67	5	97.08	9	99.83
2	75.66	6	98.56	10	99.91
3	87.99	7	99.29	11	99.96
4	94.08	8	99.65	12	99.98

**Table 4:** Starting and ending times for different double-confirmation proportions.

Proportion of double confirmation (%)	Starting time	Ending time
90	3 h 15 min	3 h 55 min
95	4 h 14 min	4 h 34 min
98	5 h 32 min	5 h 40 min

## Data Availability

The data underlying the results presented in the study are available within the manuscript.

## References

[1] Jin L. (2003). *Urban Disaster Defense and Integrated Crisis Management*.

[2] Wang Y., Wang Z. (2008). Establishment of early warning system for public health emergencies and discussion of countermeasures. *Chinese Journal of Public Health*.

[3] (2019). *Student Information Management System Based on Cloud Computing*.

[4] Zhou X. (2020). *Study of Emergency Information Management Issues in COVID-19 Pandemic Prevention and Control, and Countermeasures*.

[5] Ma F., Song E. (2011). *Basics of Information Management*.

[6] Qian D., Zhang X. (2010). A growth model for SNS. *Journal of Hefei University of Technology (Natural Science)*.

[7] Wang Y. (2014). The metric model of information dissemination based on social network. *Software Guide*.

[8] Su X., Jiang X. (2020). Function and value of a new information system for rapid response to emergency: taking prevention of COVID-19 for example. *Library & Information*.

[9] Xue J., Zhuang J., Liang F. (2006). Information management in vocational education. *Chinese Vocational and Technical Education*.

[10] Pan M., Song W. (2016). *Information Resource Database Building at Vocational Colleges Based on Big Data*.

[11] Zhang M. (2012). Thinking on strengthening the IT building of vocational education resources. *Vocational and Technical Education*.

[12] Trustdata (2019). Analysis report of the chinese mobile internet industry during january-september 2019.

[13] Tang Y., Ma Y. (2006). Information communication in small-world social networks. *Journal of System Simulation*.

[14] Li Y., Wang S. (2020). Identifying features of related information release when facing public health emergency. *Library & Information*.

